The article "Genetic Variants in DNA Double-Strand Break Repair Genes and Risk of Salivary Gland Carcinoma: A Case-Control Study" was retracted in 2018. Reasons: fabricated or falsified data; an official misconduct investigation; misconduct by an author; ethical violations by an institution or third party.

# Genetic Variants in DNA Double-Strand Break Repair Genes and Risk of Salivary Gland Carcinoma: A Case-Control Study

**DOI:** 10.1371/journal.pone.0128753

**Published:** 2015-06-02

**Authors:** Li Xu, Hongwei Tang, Adel K. El-Naggar, Peng Wei, Erich M. Sturgis

**Affiliations:** 1 Department of Head and Neck Surgery, The University of Texas MD Anderson Cancer Center, Houston, Texas, United States of America; 2 Department of Gastrointestinal Medical Oncology, The University of Texas MD Anderson Cancer Center, Houston, Texas, United States of America; 3 Department of Pathology, The University of Texas MD Anderson Cancer Center, Houston, Texas, United States of America; 4 Division of Biostatistics and Human Genetics Center, School of Public Health, The University of Texas Health Science Center, Houston, Texas, United States of America; 5 Department of Epidemiology, The University of Texas MD Anderson Cancer Center, Houston, Texas, United States of America; St. Georges University of London, UNITED KINGDOM

## Abstract

DNA double strand break (DSB) repair is the primary defense mechanism against ionizing radiation-induced DNA damage. Ionizing radiation is the only established risk factor for salivary gland carcinoma (SGC). We hypothesized that genetic variants in DSB repair genes contribute to individual variation in susceptibility to SGC. To test this hypothesis, we conducted a case-control study in which we analyzed 415 single nucleotide polymorphisms (SNPs) in 45 DSB repair genes in 352 SGC cases and 598 controls. Multivariate logistic regression analysis was performed to calculate odds ratios (ORs) and 95% confidence intervals (CIs). Rs3748522 in *RAD52* and rs13180356 in *XRCC4* were significantly associated with SGC after Bonferroni adjustment; ORs (95% CIs) for the variant alleles of these SNPs were 1.71 (1.40-2.09, *P*=1.70 × 10^-7^) and 0.58 (0.45-0.74, *P*=2.00 × 10^-5^) respectively. The genetic effects were modulated by histological subtype. The association of *RAD52*-rs3748522 with SGC was strongest for mucoepidermoid carcinoma (OR=2.21, 95% CI: 1.55-3.15, *P*=1.25 × 10^-5^, *n*=74), and the association of *XRCC4*-rs13180356 with SGC was strongest for adenoid cystic carcinoma (OR=0.60, 95% CI: 0.42-0.87, *P*=6.91 × 10^-3^, *n*=123). Gene-level association analysis revealed one gene, *PRKDC*, with a marginally significant association with SGC risk in non-Hispanic whites. To our knowledge, this study is the first to comprehensively evaluate the genetic effect of DSB repair genes on SGC risk. Our results indicate that genetic variants in the DSB repair pathways contribute to inter-individual differences in susceptibility to SGC and show that the impact of genetic variants differs by histological subtype. Independent studies are warranted to confirm these findings.

## Introduction

Salivary gland carcinoma (SGC) accounts for only 0.3% of all malignancies in the United States [1]. Although some exposures have been proposed to contribute to salivary gland carcinogenesis, including smoking [2, 3], alcohol drinking [3, 4], hormonal factors [5], and dietary factors [6], the only well-established risk factor is exposure to ionizing radiation (IR). Several studies have shown significantly increased risks of SGC among atomic bomb survivors and patients who have undergone radiotherapy for various diseases of the head and neck [7, 8]. One of the major subtypes of SGC is mucoepidermoid carcinoma[9]. Like the frequency of SGC, the frequency of the mucoepidermoid carcinoma subtype has been reported to be disproportionately high among atomic bomb survivors [7]. Intriguingly, about 80% of mucoepidermoid carcinomas are characterized by the t(11q21, 19p13) translocation [9]. Translocation occurs due to DNA double-strand breaks (DSBs), the most serious form of DNA damage caused by IR. However, only a very small proportion of individuals exposed to IR ultimately develop SGC, suggesting that there is a range of susceptibility to IR-induced salivary gland carcinogenesis. These observations underscore the crucial role of the defense system again DNA DSBs in salivary gland carcinogenesis and led us to hypothesize that inherited variants in DSB repair pathway genes contribute to individual variation in susceptibility to SGC.

To test our hypothesis, we evaluated the association of common genetic variations in 45 genes composing the DSB repair pathways with risk of SGC in 352 patients with SGC and 598 cancer-free controls. We analyzed both SNP-level and gene-level associations. In addition, we performed stratification analysis by age, sex, race, and other possible risk factors to study possible gene-environment interactions. We found that variant alleles of two SNPs were associated with SGC, and the associations were modified by histological subtype of SGC.

## Materials and Methods

### Study population

The study was approved by the Institutional Review Board at The University of Texas MD Anderson Cancer Center, and all participants provided written informed consent before inclusion in the study. The case-control study included 352 SGC cases and 598 controls prospectively recruited between 2001 and 2014 at MD Anderson Cancer Center. The cases were patients diagnosed with SGC by pathological examination, and the controls were recruited from among unrelated visitors to the institution. Recruitment criteria included age of 18 years or older, no prior malignancy except nonmelanoma skin cancer, no blood transfusion in the past 6 months, and not taking immunosuppressant medications at the time of recruitment. All study participants were US residents. Each participant donated 20 ml of peripheral blood and completed a self-administrated questionnaire covering demographic and exposure factors. Race/ethnicity was categorized as non-Hispanic white and other. Ever-smokers were defined as individuals who had smoked more than 100 cigarettes in their lifetime, and ever-drinkers were defined as individuals who had used alcohol at least once a week for more than 1 year. Body mass index was calculated from self-reported height and weight at recruitment and categorized as underweight or normal weight (<25.0 kg/m^2^), overweight (25.0–29.9 kg/m^2^), or obese (≥30 kg/m^2^) according to the World Health Organization definition.

### Genotyping and gene and SNP selection

Genomic DNA extracted from peripheral blood was used for genotyping. The DNA concentration of each sample was measured by using a NanoDrop spectrophotometer (Thermo-Fisher, Wilmington, DE) and confirmed by using PicoGreen assay (Life Technologies, Carlsbad, CA). Qualified DNA samples were then genotyped using Illumina HumanCoreExome Beadchips (Illumina, SanDiego CA). The genotyping was performed on the Illumina iScan system at the Sequencing and Microarray Facility at MD Anderson Cancer Center, where the individuals performing the assay were blinded to case-control status.

After quality-control filtering, in which low-quality SNPs and uncommon variants (minor allele frequency <5%) were removed, the remaining SNPs were annotated by using the UCSC genome browser data retrieval tool and assigned to genes on the basis of a 20-kb window on either side of the gene region defined by the human genome database version 19 [10]. Lists of genes in the DNA DSB repair pathways were obtained from the NCBI Biosystem database [11]. Overall, 415 SNPs in 45 genes in DNA DSB repair pathways were annotated and selected for association analysis.

### Statistical analysis

Demographic and exposure variables were compared between cases and controls using the chi-square test. An unconditional logistic regression model was used to derive odds ratios (ORs) and 95% confidence intervals (CIs) of SGC risk at the SNP level, with adjustment for age, sex, race/ethnicity, obesity status, and radiotherapy history. The additive model of inheritance was employed in all SNP-level association analyses. The threshold of significance level was set at a *P* value of 1.20 × 10^–4^, corresponding to Bonferroni correction for multiple tests (415 SNPs). The analysis of SNP-level association was further stratified by age, sex, race/ethnicity, smoking, alcohol drinking, first-degree family history of cancer, and obesity status to evaluate possible interactions between these variables and selected SNPs. The significance of interactions was evaluated with a likelihood ratio test that compared the fit of the full model with the interaction term versus the main effect model. Histological subtype-specific association analysis was also performed using multivariate multinomial logistic regression model. A *P* value of < 4.0 × 10^–5^ was considered significant in the subtype-specific association analysis after Bonferroni correction (415 SNPs and multiple comparisons between subtypes and controls). The statistical analysis was performed using SAS software, version 9.2 (SAS Institute, Cary, NC). All statistical tests were two-sided.

Association analysis at the gene level was performed using the logistic kernel machine (LKM) test [12]. The logistic kernel machine model integrates a logistic regression model with a semidefinite linear kernel function and takes into account the joint effect of the set of SNPs belonging to the same gene/region to test gene-disease association [13]. The gene-level association analysis controlled for age, sex, radiotherapy history, smoking, alcohol drinking, family history of cancer, obesity status, and five principal components. The threshold of significance for the logistic kernel machine test was set at 1.11 × 10^–3^ (Bonferroni correction of 0.05/45). The statistical analysis was performed using R software, version 3.1.0.

## Results

Characteristics of the cases and controls are summarized in Table 1. The majority of participants were non-Hispanic white. Cases were significantly more likely than controls to report a history of radiotherapy (2.9% vs. 0.5%), but the vast majority of the participants did not have such a history. Cases were more likely than controls to be obese (36.2% vs. 17.4%) but were less likely than controls to be an ever-drinker (49.9% vs. 57.5%) and to report a first-degree family history of cancer (53.1% vs. 61.7%). The most common histological subtypes were adenoid cystic carcinoma (35.0%), mucoepidermoid carcinoma (21.1%), and adenocarcinoma or salivary duct carcinoma not otherwise specified (14.2%). Histological subtype-specific association analysis was subsequently performed in these subtypes.

**Table 1:** Characteristics of the study subjects at recruitment.

Characteristic	Cases (n = 352)		Controls (n = 598)		
	n	%	n	%	*P*
Sex					
Male	157	44.6	233	39.0	0.088
Female	195	55.4	365	61.0	
Age, years					
≤50	139	39.5	268	44.8	0.109
>50	213	60.5	330	55.2	
Race/ethnicity					
Non-Hispanic white	266	75.6	453	75.8	0.949
Others	86	24.4	145	24.2	
Smoking					
Never	193	55.1	336	56.5	0.691
Ever	157	44.9	259	43.5	
Alcohol drinking status					
Never	175	50.1	253	42.5	0.023
Ever	174	49.9	342	57.5	
Radiotherapy history					
Yes	10	2.9	3	0.5	0.006
No	339	97.1	587	99.5	
First-degree family history of cancer					
Yes	186	53.1	367	61.7	0.010
No	164	46.9	228	38.3	
Body mass index					
Normal weight or underweight	90	26.5	256	45.5	<0.001
Overweight	127	37.3	209	37.1	
Obese	123	36.2	98	17.4	
Histological subtype					
Adenoid cystic carcinoma	123	35.0			
Mucoepidermoid carcinoma	74	21.1			
Adenocarcinoma or salivary duct carcinoma not otherwise specified	50	14.2			
Acinic cell carcinoma	40	11.4			
Other	64	18.2			

The minor allele frequencies and corresponding risk estimates for the top eight SNPs associated with SGC risk are presented in Table 2. Of these top eight SNPs, four were located within the *XRCC4* gene region. Three *XRCC4* SNPs (rs6452524, rs6452526, rs2662242) were in linkage disequilibrium but were independent of *XRCC4*-rs13180356 (r^2^<0.25). Two SNPs were significantly associated with SGC risk after Bonferroni adjustment (*P*<1.20 × 10^–4^): rs3748522 in *RAD52* and rs13180356 in *XRCC4*; ORs (95% CIs) for the variant alleles of these SNPs were 1.71 (1.40–2.09) and 0.58 (0.45–0.74), respectively.

**Table 2:** Top SNPs exhibiting significant association with risk of salivary gland carcinoma.

				MAF			
SNP	Candidate gene	Chromosome	Allele	Case	Control	OR (95% CI)	*P* ^1^
rs3748522	*RAD52*	12	C>A	0.51	0.38	1.71 (1.40–2.09)	1.70 × 10^−7^
rs13180356	*XRCC4*	5	G>A	0.19	0.28	0.58 (0.45–0.74)	2.00 × 10^–5^
rs6452524	*XRCC4*	5	G>A	0.47	0.36	1.42 (1.17–1.73)	3.62 × 10^–4^
rs6452526	*XRCC4*	5	G>A	0.47	0.37	1.40 (1.16–1.70)	5.31 × 10^–4^
rs2662242	*XRCC4*	5	A>G	0.46	0.37	1.37 (1.13–1.67)	1.58 × 10^–3^
rs1859604	*RPA3*	7	C>A	0.34	0.40	0.72 (0.58–0.90)	4.11 × 10^–3^
rs12334811	*PRKDC*	8	G>A	0.11	0.16	0.59 (0.43–0.81)	1.31 × 10^–3^
exm810950	*DCLRE1C*	10	A>G	0.17	0.12	1.55 (1.18–2.05)	1.90 × 10^–3^

MAF, minor allele frequency.

^1^Adjustment for age, sex, race/ethnicity, radiotherapy history, and obesity status.

We further performed stratification analyses exploring possible interactions between each of these two SNPs and stratified variables (Table 3). The association of *RAD52*-rs3748522 with SGC was stronger among women (OR = 2.00, 95% CI: 1.53–2.62) than among men (*P* for interaction = 0.085). *XRCC4*-rs13180356 showed significant interaction effects with sex and age; the association with SGC risk was much stronger among women (OR = 0.39, 95% CI: 0.27–0.56) than among men and much stronger among individuals ≤50 years old (OR = 0.40, 95% CI: 0.26–0.61) than among older individuals. The association of *XRCC4*-rs13180356 with SGC risk was also stronger among ever-drinkers, individuals who reported a first-degree family history of cancer, and nonobese individuals; these interactions were marginally significant. The association of *RAD52*-rs3748522 with SGC was strongest for the mucoepidermoid carcinoma subtype (OR = 2.21, 95% CI: 1.55–3.15), reaching Bonferroni-adjusted significance; the association of *XRCC4*-rs13180356 with SGC was strongest for the adenoid cystic carcinoma subtype (OR = 0.60, 95% CI: 0.42–0.87).

**Table 3:** Stratification analysis for associations between the SNPs XRCC4- rs13180356 and RAD52- rs3748522 and risk of salivary gland carcinoma.

	*XRCC4*-rs13180356		*RAD52*-rs3748522	
Stratification variable	OR (95% CI)^1^	*P*	OR (95% CI)^1^	*P*
Sex				
Male	0.87 (0.61–1.24)	0.44	1.36 (1.01–1.84)	0.047
Female	0.39 (0.27–0.56)	5.30 × 10^–7^	2.00 (1.53–2.62)	5.36 × 10^–7^
*P* for interaction		0.003		0.085
Age, years				
≤50	0.40 (0.26–0.61)	1.54 × 10^–5^	1.78 (1.31–2.41)	2.10 × 10^–4^
>50	0.72 (0.52–0.99)	0.044	1.70 (1.29–2.23)	1.38 × 10^–4^
*P* for interaction		0.025		0.71
Race/ethnicity				
Non-Hispanic white	0.69 (0.53–0.91)	9.11× 10^–3^	1.59 (1.26–2.00)	8.64 × 10^–5^
Smoking				
Never	0.55 (0.39–0.77)	4.66 × 10^–4^	1.78 (1.36–2.32)	2.63 × 10^–5^
Ever	0.61 (0.42–0.90)	0.013	1.67 (1.23–2.28)	1.21× 10^–3^
*P* for interaction		0.82		0.63
Alcohol drinking status				
Never	0.78 (0.54–1.12)	0.18	1.47 (1.09–1.98)	0.012
Ever	0.47 (0.33–0.67)	2.87 × 10^–5^	1.88 (1.42–2.48)	8.24 × 10^–6^
*P* for interaction		0.054		0.29
First-degree family history of cancer				
Yes	0.69 (0.49–0.96)	0.028	1.77 (1.35–2.32)	4.23 × 10^–5^
No	0.44 (0.30–0.65)	4.37 × 10^–5^	1.87 (1.36–2.55)	9.49 × 10^–5^
*P* for interaction		0.079		0.76
Obesity status				
No	0.49 (0.36–0.66)	3.59 × 10^–6^	1.72 (1.36–2.17)	4.45 × 10^–6^
Yes	0.93 (0.58–1.49)	0.77	1.62 (1.08–2.45)	0.021
*P* for interaction		0.051		0.88
Histological subtype				
Adenoid cystic carcinoma	0.60 (0.42–0.87)	6.91× 10^–3^	1.41 (1.06–1.87)	0.017
Mucoepidermoid carcinoma	0.57 (0.36–0.92)	0.020	2.21 (1.55–3.15)	1.25 × 10^–5^
Adenocarcinoma or salivary duct carcinoma	0.84 (0.49–1.41)	0.49	1.61 (1.04–2.51)	0.033

^1^Adjustment for age, sex, race/ethnicity, radiotherapy history, and obesity status.

The gene-level association analysis in non-Hispanic whites (Table 4) showed that five genes were associated with risk of SGC at crude *P*<0.05, but only *PRKDC* was marginally significant at Bonferroni-adjusted significance level after adjustment (*P* = 0.0014).

**Table 4:** Top DNA double-strand break repair genes associated with salivary gland carcinoma in non-Hispanic whites.

Gene	No. of SNPs	Adjusted *P* ^1^	Crude *P*
*PRKDC*	3	0.0014	0.00048
*RPA3*	17	0.018	0.037
*NHEJ1*	16	0.029	0.55
*RAD50*	7	0.035	0.013
*SHFM1*	4	0.045	0.0035

^1^Adjustment for age, sex, radiotherapy history, smoking, alcohol drinking, family history of cancer, obesity status, and five principal components.

## Discussion

DNA DSB repair is a complex process that requires multiple proteins, and deficiencies in DSB repair can cause genomic instability and increase sensitivity to IR-induced carcinogenesis [14]. There are two DSB repair pathways, homologous recombination (HR) and nonhomologous end joining (NHEJ) [15]. HR requires a template with homologous sequence for accurate repair of the damaged strand, whereas in NHEJ, broken ends of stands are repaired with little or no requirement for sequence homology. The main proteins involved in these two pathways are distinct. In the present study, we investigated the association of SGC risk with DNA DSB repair genes in these two pathways using multiple analyses, from single-SNP association test to SNP-environment interaction test to gene-level association test. We believe that this study is the first to comprehensively evaluate the genetic effect of DNA DSB repair genes on SGC risk.

The analysis of 415 SNPs in 45 DNA DSB repair genes revealed that two SNPs were significantly associated with SGC risk after Bonferroni correction, which suggests that these SNPs or the variants with which these SNPs are in linkage disequilibrium may have a role in salivary gland carcinogenesis. The variant allele (A) of SNP rs3748522, located in the intronic region of *RAD52*, was associated with increased risk of SGC. The protein product of *RAD52* is a core component in the HR pathway and is also essential for single-stranded annealing and mitotic recombination [16]. The variant allele (A) of SNP rs13180356, located in the intronic region of *XRCC4*, was associated with decreased risk of SGC. The protein product of *XRCC4* is required for NHEJ, acting as a scaffolding protein to facilitate the recruitment of other NHEJ proteins to the break ends [17]. Interestingly, subgroup analysis showed that the association of *RAD52*-rs3748522 with SGC risk was the strongest in mucoepidermoid carcinoma, whereas the association of *XRCC4*-rs13180356 with SGC risk was the strongest in adenoid cystic carcinoma. It is well known that mucoepidermoid carcinoma and adenoid cystic carcinoma differ remarkably in histological differentiation, clinical behavior, and mutation profile [18, 19]. Our finding that histological subtype modified these associations of SNPs with SGC risk supports the observed difference and, if confirmed, could indicate etiological significance.

We found that *XRCC4*-rs13180356 was associated with SGC risk in women but not men; also, the interaction of this SNP with age was significant. Similarly, the association between *RAD52*-rs3748522 and SGC risk was more evident in women, although the interaction effect was not significant (*P* for interaction = 0.085). Results of an early study suggest that men are less sensitive than women to the influence of age-related decline of DNA DSB repair capacity [20]. More recent studies have begun to show that many genes and chromosomal regions, on both autosomes and sex chromosomes, exhibit sex-specific differences in gene expression [21, 22] and likely contribute differentially to complex diseases [23]. Accordingly, although evidence linking these significant SNPs with sex is missing, a sex-specific differential association between DSB repair genes and risk of SGC is plausible.

The gene-level association analysis revealed a borderline significant gene, *PRKDC*. This gene encodes the catalytic subunit of the DNA-dependent protein kinase, which has been implicated in NHEJ, V(D)J recombination, modulation of chromatin structure, and telomere maintenance. Recent findings suggest that DNA-dependent protein kinase is also able to regulate HR and thereby play a critical role in determining which mechanism (HR or NHEJ) is chosen by the cell to repair a DSB [24, 25].

This study has both strengths and limitations. We took advantage of the large-scale genotyping data and explored almost all known DSB repair genes. We applied stringent statistical analyses to screen for SNPs and genes associated with SGC risk, with an expected false-positive rate smaller than 5%. However, given that the most significant SNPs were intronic SNPs, it is unlikely that these SNPs are causal SNPs driving the association; future functional studies should be carried out to identify the “real” functional SNPs. Among the limitations of the study is the relatively small sample size, especially for stratification analysis, even though to our knowledge this is the largest study of SGC so far. In addition, limitations inherent in the case-control study design and self-reported questionnaire variables could introduce bias in the association analysis. Bias due to selection of controls from hospital visitors may have occurred given the observation of larger proportion of subjects with family history of cancer in the control group than in the case group. We performed comparison analysis of minor allele frequency between controls with and without family history of cancer and found no significant difference (results not shown), which suggests that selection bias unlikely explains the risk associations.

In summary, our data indicate that genetic variants in the DSB repair pathways contribute to variation in susceptibility to SGC and show that the impact of genetic variants differs by histological subtype. However, more studies are needed to validate these findings in larger populations and populations with different racial/ethnic backgrounds.
